The article "A Human Resource Demand Forecasting Method Based on Improved BP Algorithm" was published in 2022. Journal: Comput Intell Neurosci.

# A Human Resource Demand Forecasting Method Based on Improved BP Algorithm

**DOI:** 10.1155/2022/3534840

**Published:** 2022-03-29

**Authors:** Xingguang Lu

**Affiliations:** Henan Polytechnic University, Jiaozuo 454003, China

## Abstract

Human resources are the first resource for enterprise development, and a reasonable human resource structure will increase the effectiveness of an enterprise's human resource input and output. The reality is that even if an enterprise designs a human resource allocation plan in accordance with the corporate strategy, it is impossible for the enterprise to operate in full accordance with the plan during the operation process, so the human resource allocation plan only reflects the law of the enterprise's human resource needs during the enterprise development process. Giving effective guidance to the specific work of human resources is difficult. It is impossible to carry out effective human resources structure adjustment to adapt to changes in human resources demand due to changes in corporate tactics, business, scale, and other factors, especially when the current domestic human resources market has not yet fully formed. This paper examines the impact of key factors such as the company's business growth scale and production efficiency improvement on human resource needs with the goal of improving team structure, optimizing staff allocation, controlling labor costs, and improving efficiency and benefits. In this paper, we attempt to develop a human resource demand forecasting model based on business development and economic benefits and guided by intensive human resource development. We analyze and forecast the enterprise's total human resource employment, personnel structure, and quality structure using this model. In light of this, this paper employs an improved BP neural network to construct a human resource demand forecasting system, resulting in a new quantitative forecasting method for human resource demand forecasting with strong theoretical significance. Simultaneously, the human resource demand forecasting system developed can enable enterprises to carry out personnel demand forecasting from the actual situation, making forecasting more applicable, flexible, and accurate, allowing enterprises to realize their strategies through reasonable human resource planning.

## 1. Introduction

We live in the information age, which is also characterized by intense competition in all areas. A large number of talents are required for the country's and society's development and progress. The “Strategy of Strengthening the Country with Talents” prioritizes talent as a key factor in the development of the country, society, and businesses, with the goal of producing hundreds of millions of high-quality workers, tens of millions of specialized talents, and a large number of top-tier innovative talents. A talent team with a reasonable echelon structure and high quality will create a new situation in which talents are produced in large numbers and best used, so that we can transform from a country with a large population to a country with strong human resources and make human resources an important part of our country's overall national strength. An enterprise, as a small society, relies on its employees as an essential resource. People play an important role in business, as indicated by the Chinese characters for enterprise. If an enterprise wants to be successful, it must pay attention to human resource management, so it is especially important for enterprises to correctly anticipate human resource development in the future. Traditional human resource management methods, however, continue to predominate in some businesses, particularly small and medium-sized businesses. The traditional practice in HR management activities such as talent training and utilization, job setting, remuneration, distribution, performance appraisal, promotion, reward, and punishment is to use accumulated surface information to implement decision-making in daily management. All decisions in human resource management are based on subjective feelings, personal experience, and corporate value systems. As a result, the organization is massive, with unequal salary distribution, ineffective performance appraisal, brain drain, and low employee satisfaction. As a result, human resource management is in a passive mode. In this case, conducting salary decision analysis to provide salary decisions for enterprises is impossible; conducting enterprise diagnosis to detect potential crises in time and provide decision support is also impossible. It is necessary to obtain a large amount of effective information in order to realize the dynamic management of people through modern human resource management or to construct the related activity system of human resource management. Traditional data analysis methods can only obtain the data's surface information. To acquire accurate intrinsic qualities and linkages, we must update the concept, examine the application of data mining theory, and apply data mining technology [1, 2] and demand forecasting technology [3, 4]. Simply described, it is the objective examination of human resource management activity to maximize the use of human resource data and information. It organizes and analyzes relevant human resource data, locates data bases for the development of human resource management and conducts in-depth mining analysis, and forecasts the results based on the data analysis, with scientifically developed human resource management techniques. The importance of data will be represented in all parts of human resource management that enhance analysis and forecasting once data mining technology is applied to the field of human resource management.

With the rapid growth of the global economy, all countries face an increasing demand for talent, and the talent pool has become a critical barometer of a country's overall national strength. According to widely held perceptions, China continues to lag behind industrialized countries in the global competition for talent. Developing a human resource strategy that is relevant for the current environment, as well as learning how to recruit, retain, and cultivate talented employees, has become an essential course for organizational development and progress. To be successful in this course, flexible human resource planning will be an essential component of your success. Enterprise human resource planning includes strategic human resource planning, which is a subset of enterprise human resource planning. In order to achieve predetermined goals and fulfill the needs of all persons involved in the development process, enterprises must anticipate the supply and demand for critical individuals in advance and devise an optimal human resource strategy to meet those demands. When it comes to the execution of appropriate human resource policies and the fulfillment of company strategic goals, business human resource planning can give essential data support. Enterprise human resource forecasting is separated into two components: demand forecasting and supply forecasting. Demand forecasting is the first component, while supply forecasting is the second. Among these, forecasting human resource demand is a prerequisite for forecasting human resource supply [5]. Only by defining the personnel requirements for future development in light of the enterprise's real situation can enterprises forecast human resource supply in a planned manner and carry out appropriate human resource planning based on supply and demand balance. Excessive forecasting of required individuals will stress the firm, while a lesser number will result in a talent deficit, impeding the enterprise's further expansion and growth. As can be seen, projecting human resource needs is the foundation for designing the accompanying operating plan.

At the moment, numerous qualitative and quantitative forecasting methods, such as the Delphi method [6], the Regression Analysis method [7, 8], and the trend extrapolation method [9, 10], have been utilized to estimate enterprise people needs, many of which are reasonably mature in foreign nations method. The study of human resources began with Professor Peter F. Drucker's book “The Practice of Management.” He defined “human resources” and emphasized the unique characteristics of human resources as a dynamic resource [11]. According to eminent academic Walker, human resource strategy is an integral aspect of business strategy, and anticipating human resource demand assists in the design and implementation of corporate strategy [12]. Purkiss began in 1974 with the historical value of manpower demand, the current value of manpower demand, and changes in enterprise production capacity. He developed a relevant model for predicting human resource demand and applied it to the British steel industry at the time, with favorable results. For the effect of [13] Rachid adapted the Markov model to an enterprise's human resource forecasting in 2013. He built an enterprise human resource forecasting model and forecasted the firm's future personnel change trend using the Markov process [14]. Many scientists have focused their attention on the application of grey theory and BP neural networks in recent years, and these scholars have conducted extensive research in a variety of domains. Lin et al. used a grey prediction model to enhance the accuracy of CMM when determining the geometric tolerance of circles [15]. Tsai et al. implemented a grey forecasting model based on grey theory to forecast staff demand in telecommunications businesses [16]. Li et al. applied a grey prediction model to an industrial production process, which increased the process's precontrol ability [17]. Chan-Ben et al. employed the Markov-Fourier grey model prediction method to forecast future data based on a set of recent data, followed by the use of Fourier series to correct for the residual error generated by the retrospective prediction model, significantly improving the method's prediction accuracy [18]. Tean-Shyan et al. devised a method for forecasting seasonal time series that is based on two forecasting models: grey theory and seasonal index. The forecasting model expresses RIS as seasonality. According to his analysis, this model surpasses the other models when it comes to forecasting accuracy, including a fuzzy seasonal model, a basic moving average model, and a simple ratio-to-moving-average model [19]. Wu et al. demonstrated that the nonhomogeneous discrete grey model's starting value selection violated both the concept of new information priority and the usage requirement for deficient information in the grey model and so developed a new grey discrete grey model with fractional accumulation. The accuracy of the forecast is greater than that of the original model [20].

In terms of BP neural network research, ParasKumar applies BP neural networks and the LM algorithm to road noise prediction, using traffic flow as an input parameter to forecast the influence of cars on road noise, with the goal of reducing road noise through vehicle flow speed management. The results indicate that the BP algorithm outperforms the LM method in terms of prediction accuracy [21]. Anucha et al. used BP neural networks and RBF neural networks to forecast fuel cell performance and obtained a high prediction accuracy, indicating that both models may be used to test commercial fuel cells' performance [22]. Ismail et al. and colleagues predicted industrial bearing load deformation using a combination of the BP neural network model and the PSO model. The prediction results indicate that the combined model is more accurate [23]. In human resource management, Huang et al. introduced BP neural networks to the enterprise human resource management information system in order to investigate how to choose senior managers more effectively and obtained favorable findings [24]. Huang et al. developed a fuzzy neural network model for human resource selection, which enabled organizations to choose talent in a novel way [25]. However, these methodologies have not gained widespread acceptance in China, where demand forecasting is primarily based on qualitative analysis. Furthermore, in their own development process, Chinese companies do not prioritize the gathering and organization of historical data about their operations, as well as the nonlinear link between indicators of human resource need and predicted results. As a result, current methodologies are unable to accurately predict the human resource requirements of Chinese companies, and this study proposes a new way for doing so. The beetle search algorithm (also known as the BAS algorithm) has outstanding accuracy. This technique is based on the notion of beetles seeking for food and is well-suited for optimizing multiobjective functions. Due to the randomness of the beetle's initial value, the algorithm is not particularly good at solving high-dimensional functions, and it is prone to falling into the local optimum [26]. To increase the predictive accuracy of the BP model, this article enhances the classic BAS algorithm and presents a new BP algorithm. The single beetle in the algorithm is enhanced in this paper into a beetle group, which reduces the algorithm's influence from the random initial value and direction of the beetle, hence preventing the algorithm from slipping into the local optimum. Additionally, conduct trials to determine the upgraded BP model's ability to forecast human resource demand.

## 2. Knowledge about Human Resource Forecasting

### 2.1. Human Resource Forecasting Related Technologies

Prediction is the scientific assessment of the future development trend and law of a prediction object using appropriate means and methods and based on the prediction object's effective historical and present information. However, because information is inherently unreliable, it will eventually result in challenges and problems with forecasting. Enterprises' human resource requirements encompass both overall and individual requirements, as well as quantitative, qualitative, and structural requirements. Demand forecasting is the process of assessing and forecasting how many people are needed, their age structure, their professional structure, their educational level structure, their professional and technical poststructure, and their skill structure in the future. In the conventional meaning, data decision-making ability refers to the capacity to make scientific decisions on data and generate value. The use of data to make decisions moves to the transformation of the data-based basis, which improves the effectiveness of human resource management and increases the business's human resource value, with the primary goal of making employee development the driving force of enterprise development.

To forecast human resource demand, the proper technical preparations must be made. To begin, assess and process anticipated target and baseline indicators. The object index is used to refer to the object of human resource demand forecasting, such as personnel demand and structure; the basis index is used to refer to the variable elements affecting demand forecasting. After establishing the index system, demand forecasting is carried out for various scenarios. Generally, human resource forecasting falls into two categories: qualitative and quantitative, with qualitative study and application coming first. Qualitative forecasting entails managers and experts with extensive experience and analytical capabilities relying on familiar business knowledge, historical data, and the current state of the enterprise, and utilizing their personal experience, analysis, and judgment abilities to forecast the enterprise's future human resource development. Make a degree of prejudgment; and then synthesize the opinions of numerous specialists in a certain format to serve as the primary basis for forecasting the future state of human resources. Qualitative forecasting encompasses a variety of techniques, including management evaluation, current situation forecasting, experience forecasting, scenario description forecasting, work research forecasting, microintegration forecasting, zero-based forecasting, driving factor forecasting, and Delphi forecasting. Quantitative forecasting primarily consists of trend forecasting, statistical forecasting, workload forecasting, labor quota forecasting, trend extrapolation forecasting, budget control forecasting, industry proportion forecasting, and benchmark forecasting.

With the advancement of data technology, quantitative research on human resource forecasting is becoming increasingly prevalent. Quantitative forecasting is the process of predicting human resource demand using historical data from businesses or a variety of elements and variables. On the basis of the relatively complete historical statistical data on human resources that enterprise managers have mastered, they use certain mathematical methods to scientifically process and organize them in order to uncover the relationships between relevant factors and variables in order to forecast the future development and changes in human resources in the enterprise. Its primary characteristic is that it makes forecasts using statistical data and mathematical models, emphasizes quantitative analysis of human resource development, and is less influenced by subjective elements.

### 2.2. Comparison of Human Resource Demand Forecasting Techniques and Methods

Demand forecasting's ultimate purpose is to determine the trend of data. While the preceding qualitative and quantitative methodologies share similar concepts and stages, their processing methods are quite different. Due to the fact that different techniques have varying application scopes and technical qualities, the method selection process has an effect on the prediction outcomes and their quality. Tables 1 and 2 compare various qualitative and quantitative approaches of demand forecasting. When forecasting enterprise human resource demand, qualitative forecasting methods are frequently influenced by expert emotion or experience; therefore, the use of quantitative methods allows for a more accurate analysis of enterprise human resource data and the formation of reasonable prediction results. Because there are frequently several factors affecting the target variable in forecasting human resource demand, the multiple linear regression forecasting approach can be used to effectively and properly anticipate the quantity of human resources in an enterprise.

## 3. Human Resource Demand Prediction Model Based on Improved BP Neural Network

An error backpropagation algorithm is used to train a multilayer feedforward neural network. When the mapping connection is ambiguous, it can learn the mapping relationship between input and output mode independently and continually alter the network threshold and weight to make it easier to do so. In order to reduce network errors, as may be seen in Figure 1, the BP neural network is depicted in this research. The input layer picks variables pertaining to the demand for human resources. Eight input layers and one output layer make up the neural network. The hidden layer is calculated by the neuron empirical formula $h=\sqrt{m+n}+a$, (*a*=1,2,…, 8). Among them, *m* and *n* are the number of input and output units of the neural network, and *a* can be chosen according to the actual test situation. By verifying the fitness function of different hidden layer BP neural networks, the number of hidden layer neurons is finally selected to be 6 to ensure the accuracy and precision of the experiment.

The randomness of the BAS algorithm's beginning value and direction makes it easy for the algorithm to fall into a local optimum; hence an improved BAS algorithm (IBAS) is presented to further increase the BAS algorithm's optimization accuracy. Improving the accuracy of the BP neural network's predictions through IBAS optimization is possible. Step-by-step instructions are as follows:

(1) To indicate the direction of each beetle in the population, create an *h*-dimensional random vector and normalize it. The following is the equation to use:
  (1) $$\begin{array}{c} b=\frac{\text{rand}\left(k,1\right)}{\left\|\text{rand}\left(k,1\right)\right\|}, \end{array}$$
rand (.) generates random numbers and *b* determines the direction of the beetle.
Using the BP neural network model, the model search dimension is *k* = *MN* + *NL* + *N* + 1 if the number of neurons in the input layer is *M* (8 in this article), output layers are *L* (1 in this article), and the hidden layer has *N* neurons. The spatial coordinates of the left and right whiskers of a single beetle are
  (2) $$\begin{array}{c} \left\{\begin{array}{c} x_{\text{ir}}=x^{t}+d^{\text{it}}b,\\ x_{\text{il}}=x^{t}-d^{\text{it}}b. \end{array}\right) \end{array}$$
After the *t*-th iteration, the right whisker of the *i*th beetle moves to *x*_*ir*_, the left whisker moves to *x*_*il*_, the distance between the *i*th beetle's left and right whiskers is *d*^*it*^, and this beetle's centroid coordinate is *x*^*t*^.
(2) Determine the left and right whisker odor strength
The odor intensity of the left and right whiskers may be estimated using the fitness function fitness, updating the positions of the left and right beetles.
  (3) $$\begin{array}{c} \left\{\begin{array}{c} x^{\text{it}+1}=x^{\text{it}}-\delta^{\text{it}}b\;\sin\;g\left(f\left(x_{\text{il}}\right)\right),\\ \text{fitness}=\frac{1}{N}\sum_{j=1}^{N}{\left(t_{\text{sim}\left(j\right)}-y_{j}\right)}^{2}. \end{array}\right) \end{array}$$
The step size factor *δ*^*it*^ corresponds to the beetle that appears in the *i*-th iteration of the *t*-th repetition. When sin  *g*(*·*) is used as the sign determination function, *t*_*sim*(*j*)_ is the output value of the *j*-th sample, and *y*_*j*_ is the actual value of the *j*-th sample, the result is the sign determination function.
(3) Calculate the factor for step size
Using the step size factor, long beetles can fine-tune their search radius. To prevent the search region from being too tiny and the local minimum value from appearing, a big beginning step size should be used. The step size is set using a linear decreasing weight, and the calculation formula is as follows:
  (4) $$\begin{array}{c} \delta^{\text{it}+1}=\delta^{\text{it}}e\left(t=0,1,\ldots ,n\right). \end{array}$$

While the step size attenuation coefficient (*e*) should be a value between [0, 1], the numerical choice of the step size factor has not been led by a complete theoretical framework to far, and 0.95 has been chosen in this study as a starting point. Multiple experiments were carried out in parallel to identify the starting step size = 3 and the number of iterations *n* = 100, both of which were equal to 100.

A random number between [−0.5, 0.5] should be assigned to each beetle in the beetle group and saved in the best A set for each insect. Bestfines A is a set that records and saves the best fitness of all beetles at the current time, based on their fitness function. Use equation to iteratively update each beetle's location (2). To keep the bestA and bestfitness A sets up to date throughout time, they should be iterated according to equation (3) to acquire the corresponding fitness function value when each update is complete. As a final step, comparing the global best fitness of the entire beetle population in the two sets yields the best beginning position of the population and the population's greatest overall fitness. Repeat the previous steps as many times as necessary. As soon as the fitness function value hits the predetermined value of 0.001 or the maximum number of iterations, bestB can be deemed the optimal initial weights and thresholds for subsequent secondary training and learning of the BP neural network at this moment. The specific procedure is shown in Figure 2.

## 4. Results and Analysis

### 4.1. Experimental Data

This study takes a mobile branch in a city as an example and forecasts the demand for human resources based on the existing data from 2005 to 2016.  Table 3 provides the specifics.

Because neural networks require all input variables to be real numbers between 0 and 1, the collected sample data must be normalized. The maximum-minimum normalization method was used in this study's processing. This method involves applying a linear transformation to the data, which can map it to the 0-1 interval. Let min and max represent the indicator *x*'s minimum and maximum values, respectively. The formula for mapping the value *v* in the indicator *x* to the 0 + 1 interval is

(5) $$\begin{array}{c} v^{\prime }=\frac{v-\min_{x}}{\max_{x}-\min_{x}}. \end{array}$$

The acquired data should be separated into training and test sets since the neural network can learn relevant knowledge. In this study, the number of samples in the training set is determined using the usual approach, and the collected samples are divided into two independent sets, which are used as the training set and the test set, respectively. Sample data from 2005 to 2014 is utilized to train the neural network, while data from 2015 and 2016 is used to test the neural network's accuracy. A new version of the BP method sets parameter *e* to 0.9. Only 500 trainings of BP neural networks can be performed, with 0.001 as the training target and learning rate.

### 4.2. Experimental Results and Analysis

Table 4 shows the experimental results after using the trained model to predict the test data.

The data in Table 4 show that the relative error is less than 7%, indicating that the neural network prediction system for human resources structure we developed is accurate. Figures 3–8 depict the results of the annual forecast of the staff-to-researcher ratio.

As a result of the research, the following conclusions can be drawn:

1. From 2005 to 2016, a neural network model was used to fit the 12-year data of a mobile company in a city, and the proportion of managers and researchers in 2015 and 2016 was predicted. According to the results, all of the errors are less than 7%, which meets the prediction accuracy requirements.
2. When compared to the linear regression model, the BP network parameter determination process is an iterative learning process, and the strong collinearity of the data frequently causes problems when performing linear regression, but it will not cause many problems in the neural network model. The BP neural network model produces weights and thresholds as results, and the interpretation of the relationship between dependent variables and independent variables in the model is not as intuitive as linear regression or time series analysis. It is difficult to predict how much an independent variable will cause the dependent variable to change in a multilayer network when other independent variables remain constant. The reason for this is that, in the linear model, the roles of the various variables can be separated, whereas in the BP network model, the influence of an independent variable on the dependent variable is dependent not only on the change of the independent variable, but also on the change of other independent variables. The variable's value: The BP network loses the intuitiveness of model interpretation in exchange for a more accurate prediction result. As a result, the neural network model outperforms the traditional human resource forecasting tool for complex nonlinear human resource structure forecasting.
3. Although the BP neural network can solve problems that traditional processing methods cannot, there is no exact theoretical guidance on how to select and determine a suitable neural network structure in practical applications. Structure of a network: At the same time, because the weights and thresholds in the BP neural network's training process are generated at random, the results of each training and prediction are different, implying that the prediction results are extremely unstable. It is necessary to repeat training, and it is only used when the multiple output results are within a certain error range.
4. Based on the data analysis, the proportion of scientific research personnel is rationalized, which is consistent with the requirement that the mobile industry research personnel team be high and precise. Year after year, the proportion of managers decreases while management efficiency improves. According to the forecast results, enterprises can optimize internal personnel and organizational structure, vigorously cultivate scientific research personnel, and maintain the team's stability. It has a significant impact on an organization's ability to effectively manage its workforce.

To summarize, any enterprise's microprediction is inextricably linked to the influence of macroeconomic trends and is constrained by the market environment. As a result, in order to make the forecast of human resource structure more realistic and practical, the changes and trends in the country's industrial policy on the industry during the forecast period, as well as the impact of the current international situation on mobile enterprises, should be taken into account in the future. The restructuring of the mobile industry, in particular, and the use of mobile 4G will exacerbate the situation. As a result, in the future, it will be necessary to continuously optimize the forecasting model's indicators in order to deal with more complex changes in human resource forecasting.

## 5. Conclusion

Human resource is the key application field of enterprise survival. With the continuous development of the enterprise, a large number of data related to human resources will be generated within the enterprise. Mining the value of these data and benefiting from it has always been a problem ignored by enterprises. This study combines the mining technology required by data mining with the demand prediction algorithm and constructs a human resource demand prediction system based on data mining. Apply the designed system to the analysis of enterprise human resource data, reveal the relationship between enterprise internal data, reveal the trend law contained in human resource data, and help enterprise decision-makers take corresponding measures. These measures determine the human capital status of enterprises, continuously improve the operation efficiency of enterprises, and finally realize the best allocation of resources. In this paper, the improved BP neural network is used as the prediction model, and its prediction accuracy is obviously improved. The optimized initial weight and threshold of BP neural network are obviously better than those in random state, which overcomes the shortcomings of BP neural network, such as slow convergence speed and easy fall into local minimum. The experimental results show that the prediction model established in this paper can accurately predict the demand of human resources. However, there are some flaws in the paper. First, the human resource demand forecasting model still has some limitations. The improved BP neural network model can be used in situations in the enterprise where the data related to personnel demand is very small or the data sequence is very volatile. The accuracy of the prediction is low. Second, pure quantitative forecasting methods can be difficult to use when dealing with rapid changes in the external environment, and forecast results are not absolute, so enterprise managers must modify forecast results through qualitative analysis.

## Figures and Tables

**Figure 1:** Improved BP neural network structure.

**Figure 2:** The improved BP neural network prediction flowchart.

**Figure 3:** Prediction results of the total output value of enterprises.

**Figure 4:** Economic benefit forecast results.

**Figure 5:** Prediction results of the total number of employees in the enterprise.

**Figure 6:** Prediction results of turnover ratio.

**Figure 7:** Predicted results of the proportion of managers.

**Figure 8:** Prediction results of the proportion of scientific researchers.

**Table 1:** Comparison of qualitative methods for demand forecasting.

Technical method main features	Technical method main features
Management evaluation	Subjective, experience has a greater impact
Current situation forecasting method	Short-term forecast, easy to operate
Experience forecasting method	Requires rich experience and objective judgment
Scenario description	Hypothetical description
Work research forecasting	Accurate job analysis is required
Microintegration	Short-term forecast, enterprise stability is required
Zero-based forecasting	Requires a thorough analysis of manpower needs
Driving factor	Find the root cause of the driving force
Delphi method	Expert independent judgment, long time

**Table 2:** Comparison of quantitative methods for demand forecasting.

Technical method main features	Technical method main features
Trend forecasting method	Single factor change
Statistical forecasting method	Statistical modeling
Workload forecasting method	Estimated workload
Labor quota method	Total tasks, labor quota
Trend extrapolation method	A clear trend over time
Budget control method	Cost budget control
Industry proportion method	Adapt to professional division of labor
Benchmark method	Follow the example

**Table 3:** Relevant data of a mobile branch in a city from 2005 to 2016.

Year	The total output value of the enterprise/100 million	Economic benefit/100 million	Total number of employees/thousands	Turnover ratio	Management ratio	Ratio of researchers
2005	9.81	1.33	2.20	4.53	3.40	61.75
2006	11.90	1.65	2.11	3.89	3.32	63.98
2007	12.13	1.83	2.05	3.96	3.29	64.32
2008	13.34	1.95	2.03	4.02	3.28	64.53
2009	14.32	2.11	2.00	4.31	3.28	65.02
2010	15.11	2.35	2.02	4.52	3.26	66.53
2011	17.20	2.52	2.04	4.32	3.25	66.46
2012	18.64	2.65	2.12	4.22	3.26	67.76
2013	19.89	2.98	2.31	4.13	3.23	66.49
2014	20.46	3.04	2.42	4.04	3.22	65.48
2015	22.54	3.25	2.35	3.68	3.20	66.33
2016	23.78	3.47	2.21	3.75	3.14	67.58

**Table 4:** Comparison of forecasts of various indicators.

Predictor	Year	True	Predicted	Relative error (%)
Total enterprise output value	2015	22.54	22.01	2.35
	2016	23.78	24.56	3.28

Economic benefits	2015	3.25	3.16	2.77
	2016	3.47	3.62	4.32

Turnover ratio	2015	3.68	3.45	6.25
	2016	3.75	3.63	3.20

Total number of employees/thousands	2015	2.35	2.22	5.53
	2016	2.21	2.16	2.26

Ratio of managers	2015	3.20	3.23	0.94
	2016	3.14	3.22	2.55

Ratio of researchers	2015	66.33	64.95	2.08
	2016	67.58	65.34	3.31

## Data Availability

The data used to support the findings of this study are available from the corresponding author upon request.
